The article "Population genetic analysis of Shaanxi male Han Chinese population reveals genetic differentiation and homogenization of East Asians" was retracted in 2024. Reasons: lack of ethics approval or compliance; missing or withdrawn patient consent; no approval from the institution; concerns about the data.

# Population genetic analysis of Shaanxi male Han Chinese population reveals genetic differentiation and homogenization of East Asians

**DOI:** 10.1002/mgg3.1209

**Published:** 2020-03-12

**Authors:** Luyao Li, Xing Zou, Guanjun Zhang, Hongyan Wang, Yongdong Su, Mengge Wang, Guanglin He

**Affiliations:** ^1^ Department of Pathology The First Affiliated Hospital of Xi'an Jiaotong University Xi'an Shaanxi China; ^2^ Institute of Forensic Medicine West China School of Basic Science and Forensic Medicine Sichuan University Chengdu Sichuan China; ^3^ Forensic Identification Center Public Security Bureau of Tibet Tibetan Autonomous Region Lhasa Tibet Tibetan Autonomous Region China

**Keywords:** forensic science, genetic differentiation, Han Chinese, population genetics, short tandem repeats

## Abstract

**Background:**

Shaanxi province, located in the upper Yellow River, has been evidenced as the geographic origin of Chinese civilization, Sino‐Tibetan‐speaking language, and foxtail or broomcorn millet farmers via the linguistic phylogenetic spectrum, archeological documents, and genetic evidence. Nowadays, Han Chinese is the dominant population in this area. The formation process of modern Shaanxi Han population reconstructed via the ancient DNA is on the way, however, the patterns of genetic relationships of modern Shaanxi Han, allele frequency distributions of high mutated short tandem repeats (STRs) and corresponding forensic parameters are remained to be explored.

**Methods:**

Here, we successfully genotyped 23 autosomal STRs in 630 unrelated Shaanxi male Han individuals using the recently updated Huaxia Platinum PCR amplification system. Forensic allele frequency and parameters of all autosomal STRs were assessed. And comprehensive population genetic structure was explored via various typical statistical technologies.

**Results:**

Population genetic analysis based on the raw‐genotype dataset among 15,803 Eurasian individuals and frequency datasets among 56 populations generally illustrated that linguistic stratification is significantly associated with the genetic substructure of the East Asian population. Principal component analysis, multidimensional scaling plots and phylogenetic tree further demonstrated that Shaanxi Han has a close genetic relationship with geographically close Shanxi Han, and showed that Han Chinese is a homogeneous population during the historic and recent admixture from the STR variations. Except for Sinitic‐speaking populations, Shaanxi Han harbored more alleles sharing with Tibeto‐Burman‐speaking populations than with other reference populations. Focused on the allele frequency correlation and forensic parameters, all loci are in accordance with the minimum requirements of HWE and LD. The observed combined probability of discrimination of 8.2201E‐28 and the cumulative power of exclusion of 0.9999999995 in Shaanxi Han demonstrated that the studied STR loci are informative and polymorphic, and this system can be used as a powerful routine forensic tool in personal identification and parentage testing.

**Conclusion:**

Both the geographical and linguistic divisions have shaped the genetic structure of modern East Asian. And more forensic reference data should be obtained for ethnically, culturally, geographically and linguistically different populations for better routine forensic practice and population genetic studies.

## Abstract 2

Population genetic analysis based on the raw‐genotype dataset among 15,803 Eurasian individuals and frequency dataset among 56 populations generally illustrated that linguistic stratification is significantly associated with the East Asian population genetic substructure. Principal component analysis, multidimensional scaling plots, and phylogenetic tree further demonstrated that Shaaxi Han has a close genetic relationship with geographically close Shanxi Han, and showed that Han Chinese is a homogeneous population during the historic and recent admixture. Except for Sinitic‐speaking populations, Shaanxi Han harbored more alleles sharing with Tibeto‐Burman‐speaking populations than with other reference populations.

## 1 INTRODUCTION

Forensic DNA profiling with sets of highly polymorphic short tandem repeat (STR) loci has become a pivotal niche in forensic investigations for nearly 30 years (Hagelberg, Gray, & Jeffreys, 1991; Kayser & de Knijff, 2011). STRs, also referred to as microsatellites, are DNA sequences containing a variable number of tandemly repeated short sequence motifs (2–6 bp) and are ubiquitously scattered throughout the eukaryotic genomes (Ellegren, 2004). STR profiling has played a key role in identifying perpetrators and missing persons, determining kinship and establishing national forensic DNA databases. During the past few decades, the increasing body of STR‐based population data has replenished different national DNA databases and facilitated data sharing. To minimize adventitious matches and improve discriminating power, the officially recommended 13‐CODIS (Combined DNA Index System) core loci were expanded to 20 STRs with the addition of 7 new loci (D1S1656, D2S1338, D2S441, D10S1248, D12S391, D19S433, and D22S1045) (Hares, 2015). For the sake of increasing the compatibility with expanded CODIS and the world's biggest DNA database ‐ Chinese National Database (CND), the Huaxia Platinum System (Thermo Fisher Scientific) covering all recommended loci in the expanded CODIS and the CND has been launched (Wang et al., 2016b, 2018). This system is a six‐dye, 25‐locus, multiplex assay that allows co‐amplification and fluorescent detection of the 23 autosomal STRs (D1S1656, D2S1338, D2S441, D3S1358, D5S818, D7S820, D8S1179, D10S1248, D12S391, D13S317, D16S539, D18S51, D19S433, D21S11, D22S1045, D6S1043, CSF1PO, FGA, TH01, TPOX, VWA, Penta D and Penta E) and Amelogenin as well as Y‐InDel (rs2032678) for sex determination. However, previous Huaxia Platinum System‐based studies have focused almost exclusively on ethnic groups (Liu, Wang, He, Wang, & Hou, 2019; Wang et al., 2016b, 2018).

The Han Chinese population, as the largest ethnic group in the world, is nonetheless underrepresented in forensic investigations to catalog the forensically genetic variants (Chen, Wu, Luo, et al., 2019; He, Wang, Liu, Hou, & Wang, 2018; He, Wang, Wang, Zou, et al., 2018). Due to its large population size, large‐scale demographic migration and population expansion facilitated by ancient agriculture, genetic admixture with adjacent ethnic groups, and substantial genetic diversity among Han Chinese had been observed in previous studies (Chen, Wu, Luo, et al., 2019; Chiang, Mangul, Robles, & Sankararaman, 2018; Gao et al., 2019; Lang et al., 2019; Stoneking & Delfin, 2010). Previous whole‐genome or uniparentally genetic studies (Gao et al., 2019; Lang et al., 2019; Li, Ye, et al., 2019; Liu et al., 2018) have shed light on a general South‐North genetic divergence among Han Chinese. Genetic evidence based on low‐coverage whole‐genome sequencing of over ten thousand Han Chinese revealed an East‐West cline (Chiang et al., 2018). Furthermore, archaeological, anthropological, lexical, and genetic findings have provided evidence that the Han Chinese could trace a common ancestry in the Yellow River basin of northern China (Blench, Sagart, & Sanchez‐Mazas, 2005; Zhang, Yan, Pan, & Jin, 2019), and the population expansions and migrations of Han Chinese were driven by the development of the Yangshao and/or Majiayao Neolithic cultures. Our previous study (Chen, Wu, Luo, et al., 2019) has investigated the forensic features, genetic diversity and phylogenetic affinity of northern Han Chinese residing in Shanxi province on the basis of 23 autosomal STRs. Nevertheless, forensic characteristics and genetic makeup of Han Chinese living in Shaanxi Province are still underrepresented. Shaanxi province, lying in central China, stretching from the Qin Mountains and Shannan in the South to the Ordos Desert in the North and comprising the Wei Valley and much of the surrounding Loess Plateau, is considered one of the early cradles of Chinese civilization. Recent archeological plant documents of the earliest staple crop domestication further demonstrated that broomcorn and foxtail millet farmers originated from Shaanxi and surrounding regions (Leipe, Long, Sergusheva, Wagner, & Tarasov, 2019). Linguistic and mitochondrial evidence further supported that this region is the cradle of the formation of Tibeto‐Burman and Sinitic‐speaking populations (Li, Tian, et al., 2019; Zhang et al., 2019). The current capital of Shaanxi province—Xi'an, is one of the four great ancient capitals of China and is the eastern terminus of the Silk Road. Hence, Shaanxi Province plays a significant role in the peopling of Neolithic populations and the dissection of genetic variations of Han Chinese settling in Shaanxi province is indispensable for uncovering the origin, migration, expansion, and admixture of the Han Chinese population.

## 2 MATERIALS AND METHODS

### 2.1 Sample preparation and DNA extraction

A batch of blood samples was collected from 630 healthy unrelated male Han Chinese individuals residing in Shaanxi province. All participators enrolled in the present study had signed the written informed consents and provided self‐declared ethnicity information. This project was endorsed by the institutional review board of the First Affiliated Hospital of Xi'an Jiaotong University and carried out in accordance with the recommendations of the Declaration of Helsinki (Nicogossian, Kloiber, & Stabile, 2014). Human genomic DNA was isolated by applying the QIAamp DNA Mini Kit (Qiagen) according to the manufacturer's guidelines and the quantity of DNA template was estimated using the Nanodrop‐2000c (Thermo Fisher Scientific).

### 2.2 PCR amplification and profiling

All samples were typed using the Huaxia Platinum PCR amplification kit (Thermo Fisher Scientific) according to the manufacturer's instructions. Multiplex amplification was performed on a ProFlex 96‐well PCR System (Thermo Fisher Scientific) following the manufacturer's protocol. The reaction mix for each sample was prepared in 25 μl volume containing 10 μl of the master mix, 10 μl of primer set, 1 μl of DNA template and 4 μl of deionized water. We employed the following thermal cycler conditions: pre‐denaturation for 1 min at 95°C, followed by 26 cycles of 94°C for 3 s, 59°C for 16 s, 65°C for 29 s, then a final extension at 60°C for 5 min, and holding at 4°C. The PCR products were electrophoresed and detected on the Applied Biosystems 3500XL Genetic Analyzer (Thermo Fisher Scientific) using POP‐4 polymer. The genotype profiles were obtained by comparing with the matching allelic ladder via GeneMapper ID‐X v.1.4 (Thermo Fisher Scientific).

### 2.3 Quality control

This study was conducted in an ISO 17025 accredited laboratory, which has also been accredited by the China National Accreditation Service for Conformity Assessment (CNAS). The experiment was carried out in strict accordance with the recommendations proposed by the International Society for Forensic Genetics (ISFG) (Schneider, 2007). Laboratory internal standards and manufacturer's protocols were strictly abided to minimize errors. Negative control (ddH_2_O) and positive control (Control DNA 007) were genotyped for each batch of genotyping.

### 2.4 Dataset composition

We first merged our 630 raw genotypes of 20 overlapping STRs among different commercial STR amplification kits with 15,173 genotypes from 19 Eurasian populations (six Turkic‐speaking populations [Chen, Zou, Wang, Wang, & He, 2019; Chen, Zou, Wang, Gao, Su, et al., 2019; Jin et al., 2017; Liu et al., 2019]: Urumqi Uyghur, Hotan Uyghur, Kumul Uyghur1, Xinjiang Uyghur, Artux Uyghur, and Akto Kyrgyz; five Han Chinese populations [Chen, Zou, Wang, Gao, Su, et al., 2019; He, Wang, Liu, et al., 2018; He, Wang, Wang, Zou, et al., 2018; Liu et al., 2019; Wang et al., 2018]: Zhujiang Han, Shanxi Han, Chengdu Han, Wuzhong Hui, and Hainan Han; four Tibeto‐Burman‐speaking populations [Liu et al., 2019; Wang et al., 2018]: Liangshan Tibetan, Chengdu Tibetan, Tibet Tibetan, and Liangshan Yi; four western Eurasian populations [Alsafiah, Goodwin, Hadi, Alshaikhi, & Wepeba, 2017; Chen, Adnan, Rakha, et al., 2019; Ossowski et al., 2017; Sadam et al., 2015]: Quetta Hazara, Estonian, Poland, and Saudi Arabian). We referred to this dataset as the raw‐genotype dataset. Subsequently, a dataset merging allele frequency distribution among Shaanxi Han population and other 55 worldwide populations (Almeida et al., 2015; Choi et al., 2017; Fujii et al., 2014; Gaviria et al., 2013; Guerreiro, Ribeiro, Porto, Carneiro de Sousa, & Dario, 2017; Hossain et al., 2016; Moyses et al., 2017; Ossowski et al., 2017; Park et al., 2013, 2016; Taylor, Bright, McGovern, Neville, & Grover, 2017; Wang et al., 2016a; Wu, Pei, Ran, & Song, 2017; Yang et al., 2018; Zhang, Xia, et al., 2016; Zhang, Yang, et al., 2016) was edited from the published literature (here referred as frequency dataset) based on the 20 overlapping STRs (CSF1PO, D10S1248, D12S391, D13S317, D16S539, D18S51, D19S433, D1S1656, D21S11, D22S1045, D2S1338, D2S441, D3S1358, D5S818, D7S820, D8S1179, FGA, TH01, TPOX, and vWA).

### 2.5 Statistical analysis

We performed the exact test of Hardy‐Weinberg equilibrium (HWE) in the Arlequin with the following parameter settings: the number of steps in Markov Chin is 1,000,000 and the number of dememorization steps is 100,000. And we tested the Linkage disequilibrium between all pairs (23 autosomal STRs) of loci with the parameter settings: number of permutations: 10,000 and number of initial conditions of expectation‐maximization (EM): 2 using Arlequin 3.5 (Excoffier & Lischer, 2010). The expected heterozygosity (Ho) and expected heterozygosity (He) were also calculated using the aforementioned parameters instrumented in Arlequin 3.5 (Excoffier & Lischer, 2010). We calculated forensic allele frequency and corresponding forensic parameters, including gene diversity (GD), polymorphism information content (PIC), matching probability (PM), discrimination power (PD), typical paternity index (TPI), power of paternity exclusion (PE), and p values of Hardy–Weinberg equilibrium using the STRAF (Gouy & Zieger, 2017). We calculated the pairwise Fst genetic distance among 20 populations included in the raw‐genotype dataset using STRAF and calculated the pairwise Nei's genetic distance among 56 global populations based on the frequency dataset using the Phylip software (Cummings, 2004). Principal component analysis (PCA) based on the allele frequency distribution among 56 populations were performed using the Multivariate Statistical Package (MVSP) software 3.22 (Kovach, 2007), and we subsequently pruned the populations out of Eurasian or East Asian to explore and zoom in the patterns of genetic relationship between eastern Eurasian or East Asian. Multidimensional scaling plots among worldwide populations or East Asians were performed using our in‐house R‐script. Phylogenetic relationships among worldwide or East Asian populations were reconstructed using Mega 7.0 (Kumar, Stecher, & Tamura, 2016). Model‐based Structure analysis was carried out using STRUCTURE (Evanno, Regnaut, & Goudet, 2005).

## 3 RESULTS AND DISCUSSION

### 3.1 Allele frequency correlation and forensic parameters

We successfully genotyped 23 autosomal STRs and two sex‐determination loci in 630 unrelated Han Chinese individuals residing in Shaanxi province located in the central plain of northern China using Huaxia Platinum amplification kit. No deviations from the linkage disequilibrium were observed after Bonferroni Correction (Table S1). Allele frequency and corresponding forensic parameters of 23 autosomal STRs are presented in Table 1. All 23 autosomal STRs are in line with the Hardy‐Weinberg equilibrium. Here, a total of 271 alleles were identified in Shaanxi Han with corresponding allele frequency spanning from 0.0008 to 0.5143. TH01 harbored the smallest allele number (6), followed by TPOX (7), while Penta E possessed the largest allele number (20), followed by FGA (19). The GD values were identified ranging from 0.6436 (TH01) to 0.9170 (Penta E). GD and Ho ranged from 0.6436 to 0.9107 and 0.6238 to 0.9190, respectively. PIC values were observed spanning 0.5920 (TH01) to 0.9101 (Penta E), which is consistent with the observed minimum and maximum allele number. PM was observed ranging from 0.0146 to 0.1857 and PD spanned from 0.8143 to 0.9854. The PE values ranged from 0.3204 in the locus of TPOX and 0.8345 in the locus of Penta E. The observed individual forensic parameters of 23 autosomal STRs are suitable for choosing and applying these markers in individual identification and parentage testing, not for biogeographic ancestry inference of Shaanxi Han population. Combing the forensic effectiveness of all included loci, we identified that the combined probability of discrimination in Shaanxi Han Chinese is 8.2201E‐28 and the cumulative power of exclusion in this studied population is 0.9999999995. In accordance with the observed patterns of forensic characteristics in Chinese Turkic‐speaking, Tibeto‐Burman‐speaking and other Sinitic‐speaking populations, all included loci (23 autosomal STRs and two sex‐determinate loci) included in the Huaxia Platinum amplification kit are informative and polymorphic in Shaanxi Han Chinese population. This kit with more included STR loci than other STR kits such as the AmpFℓSTR Identifiler PCR amplification kit (He, Su, et al., 2019) (15 STRs, Thermo Fisher Scientific) is more suitable for Chinese National Database construction and forensic routine personal identification and paternity discrimination.

**Table 1:** Allele frequency distributions and corresponding forensic parameters of 23 autosomal short tandem repeats (STRs) included in the Huaxia Platinum kit in Shaanxi Han populations

Locus	CSF1PO	D10S1248	D12S391	D13S317	D16S539	D18S51	D19S433	D1S1656	D21S11	D22S1045	D2S1338	D2S441	D3S1358	D5S818	D6S1043	D7S820	D8S1179	FGA	PentaD	PentaE	TH01	TPOX	vWA
5																				0.0413			
6																			0.0024		0.0921		
7	0.0008			0.0040										0.0143		0.0016			0.0040	0.0016	0.2817		
8		0.0008		0.2373	0.0143									0.0024		0.1262	0.0024		0.0389	0.0040	0.0516	0.4841	
8.1												0.0008											
9	0.0548			0.1294	0.2921		0.0008					0.0008		0.0746		0.0667	0.0016		0.2778	0.0056	0.5143	0.1484	
9.1												0.0167				0.0063							
9.3																					0.0365		
10	0.2524			0.1619	0.1127	0.0016		0.0008				0.2611		0.2103	0.0373	0.1484	0.1111		0.1246	0.0341	0.0238	0.0286	
11	0.2349	0.0087		0.2397	0.2206	0.0024	0.0016	0.0698		0.2754		0.3635		0.2873	0.1127	0.3310	0.0786		0.1579	0.1389		0.3008	
11.3												0.0389											
12	0.3675	0.0770		0.1698	0.2270	0.0302	0.0365	0.0452		0.0048		0.1786	0.0016	0.2643	0.1286	0.2810	0.1270		0.1841	0.1024		0.0349	
12.2							0.0040																
12.3	0.0008											0.0008											
13	0.0802	0.3730		0.0532	0.1183	0.2016	0.2603	0.0992		0.0032		0.0206	0.0016	0.1270	0.1214	0.0357	0.2294		0.1563	0.0405		0.0016	
13.2							0.0333																
14	0.0056	0.2317		0.0048	0.0143	0.2175	0.2849	0.0746		0.0175	0.0008	0.1111	0.0333	0.0159	0.1302	0.0032	0.1841		0.0444	0.0881		0.0016	0.2524
14.2							0.1135																
15	0.0032	0.2024	0.0127		0.0008	0.1675	0.0659	0.3040		0.2706	0.0008	0.0071	0.3770	0.0040	0.0167		0.1786		0.0079	0.0952			0.0278
15.2							0.1373																
15.3								0.0016															
16		0.0873	0.0032			0.1294	0.0135	0.2310		0.2381	0.0103		0.3230		0.0024		0.0754	0.0008	0.0016	0.0810			0.1865
16.2							0.0460																
16.3								0.0079															
17		0.0183	0.1167			0.0810		0.0897		0.1627	0.0595		0.1960		0.0397		0.0111	0.0016		0.0873			0.2516
17.2							0.0024																
17.3			0.0008					0.0405															
18		0.0008	0.2373			0.0389		0.0103		0.0262	0.1056		0.0651		0.1897		0.0008	0.0206		0.0968			0.1865
18.2															0.0016								
18.3			0.0016					0.0190															
19			0.2357			0.0413		0.0016		0.0016	0.1452		0.0024		0.1563			0.0587		0.0683			0.0817
19.2			0.0008																				
19.3								0.0048															
20			0.1683			0.0262					0.1119				0.0444			0.0444		0.0548			0.0127
20.3															0.0008								
21			0.0817			0.0254					0.0206				0.0119			0.1087		0.0333			0.0008
21.2																		0.0008					
21.3															0.0040								
22			0.0778			0.0175					0.0484				0.0016			0.1571		0.0135			
22.2																		0.0071					
22.3															0.0008								
23			0.0365			0.0103					0.2294							0.2302		0.0079			
23.2																		0.0119					
24			0.0135			0.0040					0.1802							0.1865					
24.2																		0.0040					
25			0.0111			0.0032					0.0595							0.1135		0.0032			
25.2																		0.0063					
26			0.0024			0.0016					0.0238							0.0357		0.0024			
26.2																		0.0008					
27						0.0008			0.0016		0.0040							0.0087					
28									0.0444									0.0024					
28.2									0.0087														
29									0.2683														
29.2									0.0040														
29.3									0.0016														
30									0.2881														
30.2									0.0127														
30.3									0.0024														
31									0.1008														
31.2									0.0698														
32									0.0278														
32.2									0.1079														
33									0.0071														
33.2									0.0500														
34									0.0024														
34.2									0.0024														
Ho	0.7372	0.7528	0.8323	0.8122	0.7880	0.8555	0.8109	0.8223	0.8134	0.7673	0.8603	0.7538	0.7103	0.7818	0.8740	0.7684	0.8418	0.8561	0.8211	0.9170	0.6436	0.6516	0.7965
PIC	0.6926	0.7149	0.8106	0.7844	0.7549	0.8388	0.7859	0.8015	0.7901	0.7273	0.8445	0.7156	0.6581	0.7473	0.8600	0.7329	0.8213	0.8394	0.7968	0.9101	0.5920	0.5929	0.7647
PM	0.1096	0.1003	0.0529	0.0623	0.0771	0.0391	0.0616	0.0521	0.0603	0.0948	0.0360	0.1002	0.1455	0.0813	0.0308	0.0876	0.0462	0.0383	0.0581	0.0146	0.1857	0.1748	0.0732
PD	0.8904	0.8997	0.9471	0.9377	0.9229	0.9609	0.9384	0.9479	0.9397	0.9052	0.9640	0.8998	0.8545	0.9187	0.9692	0.9124	0.9538	0.9617	0.9419	0.9854	0.8143	0.8252	0.9268
Ho	0.7079	0.7683	0.8349	0.7905	0.7492	0.8841	0.8222	0.8063	0.8000	0.7651	0.8635	0.7286	0.7286	0.7667	0.8683	0.7429	0.8238	0.8667	0.8444	0.9190	0.6683	0.6238	0.7810
PE	0.4406	0.5415	0.6654	0.5815	0.5084	0.7631	0.6409	0.6109	0.5990	0.5359	0.7216	0.4738	0.4738	0.5387	0.7311	0.4976	0.6440	0.7280	0.6839	0.8345	0.3809	0.3204	0.5642
TPI	1.7120	2.1575	3.0288	2.3864	1.9937	4.3151	2.8125	2.5820	2.5000	2.1284	3.6628	1.8421	1.8421	2.1429	3.7952	1.9444	2.8378	3.7500	3.2143	6.1765	1.5072	1.3291	2.2826
Phwe	0.2275	0.9486	0.0222	0.1691	0.0672	0.8568	0.0157	0.3664	0.0363	0.7866	0.8095	0.0810	0.0468	0.3347	0.8005	0.0023	0.0861	0.5574	0.9014	0.3582	0.2288	0.2050	0.6677

Abbreviations: He, expected heterozygosity; Ho, observed heterozygosity; PD, discrimination power; PE, power of paternity exclusion; pHWE, p values of Hardy–Weinberg equilibrium; PIC, polymorphism information content; PM, matching probability; TPI, typical paternity index.

### 3.2 Population comparisons among Eurasian populations via raw‐genotype dataset

To explore the similarities and differences in the genetic material of Shaanxi Han population and Eurasian reference populations, pairwise Fst genetic distances among 20 populations included in the raw‐genotype dataset were calculated and presented in Table S2 and visualized in Figure 1a. Shaanxi Han population has a close genetic relationship with the geographically close Shanxi Han population with the smallest pairwise Fst genetic distance (0.0002), followed by populations belonging to the same language groups (Sinitic‐speaking Zhujiang Han: 0.0007, Chengdu Han: 0.0008 and Wuzhong Hui: 0.0009). The distant genetic relationship with Shaanxi Han in the raw‐genotype dataset was identified with the western Eurasian population (Poland: 0.0163). Turkic‐speaking populations have intermediate relationships with this studied Han Chinese population (average ± standard error: 0.0040 ± 0.0016). Patterns of genetic similarities and differences were then explored via MDS based on the top three dimensions and visualized in Figure 1b,c. Western Eurasian populations (Saudi Arabian, Poland and Estonian) were scattered than other patterns of eastern Eurasian populations. Here, we found that a close genetic affinity was identified between Hazara and Turkic‐speaking populations, which is consistent with our recent findings that the Hazara population is mixture descendants of Mongolian and local central Asians via high‐density genome‐wide data and indel markers (He, Adnan, et al., 2019). Shaanxi Han was scattered in Figure 1b and located between Chengdu Tibetan and Liangshan Tibetan in Figure 1c. These observed patterns of genetic affinity may partially reflect the common origin of Sino‐Tibetan‐speaking populations in the Upper and middle Yellow River (including the studied Shaanxi province) approximately 5,900 years before the present (Zhang et al., 2019). It should be cautious that some artifacts can be made due to the low discrimination of STR markers in population substructure exploration. Thus, to provide more genetic evidence of the similarities and differences of genetic inheritance of these populations, we reconstructed the neighbor‐joining tree in Figure 1d. Four genetic clusters can be identified in the phylogenetic relationship reconstruction result: Tibeto‐Burman‐speaking cluster, Sinitic‐speaking cluster, Turkic‐speaking cluster, and western Eurasian cluster. Here, we observed that Shaanxi Han was localized in the intermediate position between Tibeto‐Burman‐speaking populations and Sinitic‐speaking populations.

**Figure 1:** The genetic affinity between Shaanxi Han and 19 Eurasian reference populations based on the raw‐genotype data. (a) Heatmap of the pairwise Fst genetic distance. (b and c) Genetic relationship patterns among 20 populations inferred from genetic distance matrix based on the top three dimensions. (d) Phylogenetic relationship reconstruction revealed the genetic affinity between Shaanxi Han and both Sinitic and Tibeto‐Burman‐speaking populations. (e) Model‐based Structure results showed the individual and population ancestry proportion of Shaanxi Han and other reference populations

Individual and population ancestry composition was dissected via model‐based Structure analysis among 15,803 individuals (Figure 1e). At k = 2, all individuals were assigned two predefined ancestries: AntiqueWhite ancestry represented as western Eurasian ancestry and LightSkyBlue ancestry represented as eastern Eurasian ancestry. LightSkyBlue ancestry was maximized in Chengdu Tibetan (0.978) and AntiqueWhite ancestry was maximized in Poland (0.977). Turkic‐speaking populations can be modeled as mixture of one population associated with European ancestry and one population‐linked with east Asian (Xinjiang Uyghur (0.477; 0.523), Urumqi Uyghur (0.487; 0.513), Kumul Uyghur1 (0.508; 0.492), Hotan Uyghur (0.53; 0.47), Akto Kyrgyz (0.571; 0.429), Artux Uyghur (0.593; 0.407)). These patterns of European‐Asian admixture were further supported our previous findings of the mixed formation of modern Turkic‐speaking populations via ancestry‐informative markers (He, Wang, Wang, Luo, et al., 2018) and the previous genome‐wide survey of northern and southern Uyghurs via Xu, Huang, Qian, and Jin (2008). At k = 3, two predefined ancestries enriched in Han Chinese populations were observed (LightSkyBlue ancestry only enriched in Han Chinese populations and maximized in Zhujiang Han:0.495; and ForestGreen ancestry enriched in all eastern Asians and maximized in Liangshan Tibetan: 0.903 and Chengdu Tibetan: 0.868). Here, we can define LightSkyBlue ancestry as Han‐dominant ancestry and ForestGreen ancestry as Tibetan‐dominant ancestry. The third AntiqueWhite ancestry is representative of European ancestry, which was maximized in Poland (0.871). We can model Shaanxi Han as a mixture of 0.752 Liangshan Tibetan‐related ancestry, 0.231 Zhujiang Han‐related ancestry and only 0.017 Poland‐related ancestry. At k = 4 or 5, two new ancestries maximized in Saudi Arabian and Turkic populations were identified.

### 3.3 Comprehensive genetic relationship among worldwide populations via frequency‐dataset

To further investigate the genetic homogeneity and heterozygosity between the Shaanxi Han population and more reference populations and dataset consisting of allele frequency distribution, we merged our allele frequency correlation with allele frequency data from 55 worldwide populations. We first carried out the principal component analysis among 56 populations based on 613 alleles of 20 autosomal STRs. The top ten components can extract 84.083% variations from the genetic variations of 56 worldwide populations. First to tenth component accounted for 32.489%, 15.532%, 10.029%, 7.900%, 6.400%, 3.544%, 2.509%, 2.064%, 1.840%, and 1.775%, respectively. Patterns of genetic relationship among 56 populations revealed by the top four components (65.951%) are showed in Figure 2. Generally, PC1 can differentiate East Asians from other populations and PC2 ~ PC4 mainly differentiate some small substructure within‐continental populations. Due to some migrant reference populations from Africa, America and Oceania were included here, no obvious population cluster could be identified. We further removed these continental populations and focused on the genetic variations of East Asians and South Asians. 88.439% variations can be extracted via the top ten components (PC1 ~ PC10 can, respectively, account for 39.334%, 11.917%, 10.210%, 6.819%, 5.258%, 4.186%, 3.246%, 3.07%, 2.427%, and 1.969%). As shown in Figure S1, PC1 can separate East Asians and Turkic‐speaking populations, and PC2 can separate South Asian Bangladeshi and Indian. PC3 and PC4 can separate Tibeto‐Burman‐speaking populations and Japonic&Koreanic populations from others, respectively. The genetic affinity between Shaanxi Han and Central Han, Shanxi Han, and Sichuan Han can be identified here. We finally excluded two South Asian populations (Bangladeshi and Indian) and carried another PCA analysis (Figure S2). A total of 88.637% variations can be revealed by the first ten components. Three clear clusters can be observed: Turkic cluster, Tibeto‐Burman cluster, and others.

**Figure 2:** Principal component analysis among 56 worldwide populations based on the allele frequency distribution. (a–d) Two‐dimensional plots respectively reconstructed based on the random combination of the top four components

Subsequently, population genetic relationships were explored via pairwise genetic distance, multidimensional scaling plots and phylogenetic relationship reconstruction. Figure 3 and Table S3 showed the pairwise Nei's genetic distances between Shaanxi Han and the other 55 worldwide reference populations. The smallest genetic distance was 0.0029 observing between Shaanxi Han and Shanxi Han, followed by 0.0031 in Central Han, 0.0059 in Guangdong Han. As expected, the largest genetic distance with Shaanxi Han was identified in South African populations (AmaZulu: 0.1794 and AmaXhosa: 0.2012), followed by the indigenous Oceanian Polynesian. Heatmap among 56 populations based on the pairwise Nei's genetic distance matrix is shown in Figure 4. The largest distances (shown as green color) were identified between Polynesian and South Asian indigenous population and the smallest genetic distances (shown as red color) were observed within‐continental populations, especially in Han Chinese populations. Heatmap also clustered Shaanxi Han with Central Han, Southern Xiamen Han, and Northern Shanxi Han. Genetic clusters further explored using Multidimensional scaling plots among 56 worldwide populations (Figure 5a) and East Asian populations (Figure 5b). East Asians were localized in the left part and Turkic speakers were located in the intermediate position between East Asians and others from Europe, Africa, America and Oceania in the worldwide two‐dimensional plots. In the East Asian two‐dimensional plots, similar patterns of genetic relationships with PCA results were observed. Shanxi Han and Central Han Chinese populations clustered tightly with Shaanxi Han. We finally built the phylogenetic relationship on the basis of the Nei's genetic distance matrix (Figure 6). Three main branches can be categorized: African and Oceanian indigenous branch, European and American branch, and East Asian Branch. We can find that populations with similar ethnic origins tend to be formed a clade. Linguistic stratification was significantly associated with population genetic substructure in East Asian, significant examples for Sinitic, Tibeto‐Burman and the Turkic language groups included here. Shaanxi Han was first clustered with southern Han Chinese populations (Sichuan Han and Central Han) and then formed a clade with Shanxi Han.

**Figure 3:** Geographic position of Shaanxi Han and other included reference populations and the pairwise Nei's genetic distance between Shaanxi Han and the reference populations. Red color means the larger genetic distance between the studied population and the targeted reference and green color denotes the smaller genetic distance

**Figure 4:** Heatmap of the pairwise Nei's genetic distance calculated based on the allele frequency distribution in the frequency dataset. Red color denotes the strong genetic affinity, dark color means mediated genetic affinity with others and green color shows the strong genetic difference with others

**Figure 5:** Multidimensional scaling plot result of populations included in the dataset2. (a) Patterns of genetic similarities and differences among all 56 worldwide populations. (b) Population genetic substructure is associated with linguistic stratification in East Asian

## 4 CONCLUSION

We provided the first batch forensic dataset of 23 STRs included in the Huaxia Platinum PCR amplification kit from the Han population residing in Shaanxi, near the Loess Plateau which was thought of as the origin of Chinese civilization and Sino‐Tibetan‐speaking populations. Comprehensive population genetic analyses based on the raw‐genotype dataset and frequency‐dataset consistently provided new insights into the population substructure of East Asians: linguistic stratification was significantly associated with population genetic substructure. Pairwise genetic distance, PCA, MDS, heat map, neighbor‐joining tree, as well as model‐based individual and population ancestry composition dissection demonstrated that Shaanxi Han harbored a close genetic relationship with the geographically close Shanxi Han, followed by other Han Chinese and Tibeto‐Burman‐speaking populations. Significant genetic homogenization was identified in Han Chinese and genetic differentiation was observed among populations belonging to different language families. Allele frequency distribution, parameters focused on forensic effectiveness indicated that forensic markers included in the Huaxia Platinum kit are highly informative and polymorphic in Shaanxi Han populations and can be used as the routine forensic practice.

**Figure 6:** Neighbor‐Joining phylogenetic tree. Similar color denotes the common geographic origin of continental populations or the same linguistic origin of East Asian populations

## CONFLICT OF INTEREST

The authors declare that the research was conducted in the absence of any commercial or financial relationships that could be construed as a potential conflict of interest.

## AUTHOR CONTRIBUTIONS

GH and LL conceived the idea for the study. GZ, HW, XZ, and MW performed or supervised the laboratory work. GH, LL, GZ, HW, XZ, and MW analyzed the data. GH, MW wrote and edited the manuscript. We would like to thank Prof. Renata Jacewicz (Department of Forensic Genetics, Pomeranian Medical University in Szczecin, Poland), Prof. Hussain M. Alsafiah (Forensic Genetics Laboratory, General Administration of Criminal Evidences, Public Security, Ministry of Interior, Saudi Arabia), Prof. I. Zupanič Pajnič (Institute of Forensic Medicine, Faculty of Medicine, University of Ljubljana) for sharing the raw genotype data as our reference data.

## ETHICS STATEMENT

This study was approved by the First Affiliated Hospital of Xi'an Jiaotong University. This study followed the recommendations of the World Medical Association Declaration of Helsinki.

## Supporting information

Fig S1

Fig S2

Table S1

Table S2

Table S3
